RETRACTED

# Influencing Factors of Early Neurological Deterioration and Short-Term Prognosis after Intravenous Thrombolysis in Patients with Acute Ischemic Stroke

**DOI:** 10.1155/2021/6278259

**Published:** 2021-09-08

**Authors:** Guangsheng Liu, Jianghua Dai, Yinghao Ma, Yongjun Chen, Xiaohong Liao, Ao Zou, Zhian Yin

**Affiliations:** ^1^Department of Tneurology, Longhui People's Hospital, Shaoyang 422200, Hunan, China; ^2^Department of Thoracic Surgery, Longhui People's Hospital, Shaoyang 422200, Hunan, China; ^3^The Affiliated Nanhua Hospital, Department of Tneurology, Hengyang Medical School, University of South China, Hengyang 421001, Hunan, China; ^4^Department of Neurosurgery, Longhui People's Hospital, Shaoyang 422200, Hunan, China

## Abstract

**Objective:**

To explore the factors affecting the early neurological deterioration (END) and short-term prognosis of patients with acute ischemic stroke (AIS) after intravenous thrombolysis.

**Methods:**

The clinical data of 212 patients with AIS who received intravenous thrombolysis in our hospital from July 2017 to November 2020 were selected and divided into the END group (*n* = 71) and the non-END group (*n* = 141) according to the National Institute of Health Stroke Scale (NIHSS) score and divided into the poor prognosis group (*n* = 85) and the good prognosis group (*n* = 127) according to the modified Rankin scale (mRS) score at discharge. The basic data of patients, vascular risk factors, imaging examinations, and laboratory indicators were collected. A logistic regression model was used to analyze the influencing factors of END and the short-term prognosis of AIS patients after intravenous thrombolysis.

**Results:**

Univariate analysis showed that the patient's age, time from onset to treatment (OTT), NIHSS score, diabetes, hypertension, atrial fibrillation, TOAST classification, infarct size, carotid artery stenosis, white blood cell count (WBC), C-reactive protein (CRP), and D-dimer (DD) were associated with END (*P* < 0.05). Multiple logistic regression analysis found that NIHSS score, diabetes, atrial fibrillation, infarct size, carotid stenosis, and CRP were independent influencing factors of END after intravenous thrombolysis in AIS patients (*P* < 0.05). Univariate analysis showed that the patient's age, OTT, NIHSS score, diabetes, hypertension, atrial fibrillation, infarct size, carotid stenosis, and the occurrence of END were all related to the short-term prognosis of AIS patients (*P* < 0.05). Multiple logistic regression analysis showed that age, NIHSS score, infarct size, carotid artery stenosis, and the occurrence of END were all independent factors affecting the short-term prognosis of AIS patients.

RETRACTED

**Conclusion:**

High NIHSS score, combined with diabetes, atrial fibrillation, moderate to severe carotid stenosis, and elevated CRP are all risk factors for END after intravenous thrombolysis in AIS patients. Moreover, advanced age, high NIHSS score, moderate to severe carotid stenosis, and occurrence of END are risk factors for poor short-term prognosis after intravenous thrombolysis in AIS patients.

## 1. Introduction

Acute ischemic stroke (AIS) is a group of clinical syndromes in which cerebrovascular stenosis or occlusion leads to the cerebrovascular blood supply, followed by brain damage, necrosis of nerve cells, and neurological dysfunction. It is a common clinical cerebrovascular syndrome, with a significantly high rate of disability and fatality [1]. In recent years, due to the intensification of China's aging society and the changes in the lifestyles of the Chinese people, the incidence of AIS has remained high. It has become one of the most common causes of disability and death among Chinese adults, thus threatening the lives of patients [2]. At present, the main purpose of treating AIS is to improve cerebral blood circulation. The treatment methods include arteriovenous thrombolysis, intravascular intervention, and traditional Chinese medicine treatment. Among them, intravenous thrombolysis is the main treatment for AIS. Although most post-onset AIS patients tend to get better after systemic treatment, there are still some cases where the improvement is not ideal, and symptoms of progressive deterioration of neurological function appear, that is, early neurologic deterioration (END) [3]. The etiology and pathogenesis of END are complicated. At the same time, China has not yet formed a unified diagnostic standard, and there are no effective early predictive indicators, so its clinical prevention and treatment are very difficult [4]. END is closely related to the final outcome of AIS patients. If the influencing factors of END in AIS patients can be accurately assessed, and effective prevention and treatment can be carried out at the same time, it will be of great significance to reduce the disability and fatality rate of AIS [5]. This study conducted a retrospective analysis of AIS patients treated with intravenous thrombolysis and explored the impact of related factors on the occurrence of END and short-term prognosis in AIS patients after intravenous thrombolysis.

## 2. Materials and Methods

### 2.1. General Information

We retrospectively included 212 AIS patients treated with intravenous thrombolysis in our hospital from July 2017 to November 2020. Among them, 113 were males and 99 were females, aged 39–85 years, with an average age of 59.43 ± 19.77 years. All patients met the AIS diagnostic criteria in the “Chinese Guidelines for the Diagnosis and Treatment of Acute Ischemic Stroke 2014” [6] and were confirmed by head CT or MRI. All patients were treated within 4.5 hours of onset. The information of patients was complete, except for patients with cognitive dysfunction or patients with severe organ dysfunction before treatment. All patients were treated with intravenous thrombolysis by injection of alteplase (Actilyse, Boehringer Ingelheim Pharma GmbH and Co.KG, Germany) within 4.5 hours of onset, with a dose of 0.9 mg/kg and a maximum of 90 mg. First, 10% of the total dose was injected intravenously, and the remaining dose was instilled for 1 hour.

RETRACTED

### 2.2. Research Methods

Collect the following data from all patients: (1) general conditions: gender, age, onset to treatment time (OTT), and National Institute of Health Stroke Scale (NIHSS) score; (2) vascular risk factors: smoking, drinking, diabetes, hypertension, and atrial fibrillation; (3) imaging examination: TOAST classification, infarct size, degree of carotid artery stenosis, and infarct location; (4) laboratory examination: total cholesterol (TC), triglycerides (TG), low-density lipoprotein (LDL-C), high-density lipoprotein (HDL-C), homocysteine (Hcy), uric acid (UA), white blood cell count (WBC), C-reactive protein (CRP), fibrinogen (FIB), and D-dimer (DD). The NIHSS score ranges from 0 to 42 points. The higher the score, the more severe the neurological impairment of the patient. Within 7 days after treatment, if the NIHSS score increased by more than 4 points than before treatment, it was diagnosed as END. According to the results of the NIHSS score, patients were divided into 71 cases in the END group and 141 cases in the non-END group. The prognosis of patients was assessed using the modified Rankin scale (mRS) at the time of discharge from the hospital. According to the mRS score, patients were divided into a good prognosis group (mRS ≤2 points) (127 cases) and a poor prognosis group (mRS >2 points) (85 cases).

### 2.3. Statistical Methods

Data and statistical analyses were done in SPSS 22.0 software. Data plotted in linear scale were expressed as mean ± standard deviation ($\bar{x}$ ± *s*), and the *t*-test is used for pairwise comparison. The enumeration data are expressed by %, and the *χ*^2^ test is used. Multivariate analysis adopts multiple logistic regression model. The test level is *α* = 0.05, and *P* < 0.05 indicates that the difference is statistically significant.

## 3. Results

### 3.1. Single-Factor Analysis of END in AIS Patients

Univariate analysis showed that patient age, OTT, NIHSS score, diabetes, hypertension, atrial fibrillation, TOAST classification, infarct size, carotid artery stenosis, WBC, CRP, and DD were statistically significant between the END group and the non-END group difference (*P* < 0.05), as shown in Table 1.

RETRACTED

### 3.2. Analysis of Multiple Factors Affecting the Appearance of END in AIS Patients

Multivariate logistic analysis showed that the patient's NIHSS score, diabetes, atrial fibrillation, infarct size, carotid artery stenosis, and CRP were all independent influencing factors after intravenous thrombolysis in AIS patients (*P* < 0.05), as shown in Table 2.

### 3.3. Single-Factor Analysis Affecting the Short-Term Prognosis of AIS Patients

Univariate analysis showed that patient age, OTT, NIHSS score, diabetes, hypertension, atrial fibrillation, infarct size, carotid artery stenosis, and whether END occurred were statistically different between the good prognosis group and the poor prognosis group (*P* < 0.05), as shown in Table 3.

### 3.4. Analysis of Multiple Factors Affecting the Short-Term Prognosis of AIS Patients

Multivariate logistic analysis showed that patient age, NIHSS score, infarct size, degree of carotid artery stenosis, and the occurrence of END were all independent factors influencing the short-term prognosis of AIS patients after intravenous thrombolysis (*P* < 0.05), as shown in Table 4.

## 4. Discussion

In recent years, with the increase in the incidence of AIS, and due to the population bias, which mainly concentrated in the elderly with other underlying diseases, the incidence of END continues to rise, and it tends to cause a poor prognosis for AIS patients, such as disability or even death [7, 8]. The mechanism of the occurrence of END in AIS patients is not yet clear, and it is generally believed to be the result of a combination of multiple factors (such as poor medial branch circulation of the lesion, intracranial hypertension, hemorrhagic transformation, reocclusion of blood vessels); thus, it is difficult to prevent and treat END [9]. Helleberg et al. [10] showed that AIS patients with END tend to have a higher disability and fatality rate. Therefore, timely and effective assessment of various risk factors related to the occurrence of END and its short-term prognosis in AIS patients, early identification, and corresponding intervention measures are of great significance to reduce the probability of END occurrence and improve the prognosis and quality of life of AIS patients.

The results of this study showed that patient age, OTT, NIHSS score, diabetes, hypertension, atrial fibrillation, TOAST classification, infarct size, carotid artery stenosis, WBC, CRP, and DD were statistically different between END patients and non-END patients. A further multivariate logistic analysis showed that the patient's NIHSS score, diabetes, atrial fibrillation, infarct size, carotid artery stenosis, and CPR were all independent factors influencing the occurrence of END in AIS patients with intravenous thrombolysis. The possible reasons are as follows. (1) The higher the NIHSS score, the more severe the patient's condition and the larger the infarct size. Such patients are often accompanied by a variety of complications, and the free radicals produced by the complications can cause redamage of the brain tissue, leading to the occurrence of END [11, 12]. (2) Hyperglycemia itself has a toxic effect on ischemic tissues, and it can also increase the permeability of the blood-brain barrier by promoting the production of metalloproteinase-9, causing brain tissue swelling, local inflammatory cell infiltration, and aggravating nerve cells in many ways Injury, resulting in diabetic patients more likely to develop END [13, 14]. (3) Some patients with atrial fibrillation already have heart diseases such as ischemic heart disease, valvular heart disease, and sick sinus syndrome, and their heart function is weak. When combined with AIS, it is more likely to cause cardiopulmonary failure or damage to multiple organs. Studies have shown that the early mortality rate of AIS patients with atrial fibrillation is significantly higher than that of other AIS patients, which is one of the independent factors influencing the occurrence of END in AIS [15]. (4) AIS patients with excessively large infarct size and moderate to severe carotid stenosis are often difficult to establish effective collateral circulation and restore blood supply to the ischemic brain tissue, so they are more prone to irreversible damage to the ischemic penumbra. Induce END [16, 17]. (5) CRP protein is a systemic inflammatory marker. The increase in its level not only represents the activation degree of systemic inflammatory response but also promotes monocyte-macrophages to produce a large number of inflammatory factors, causing endothelial cell damage and plaque. Rupture can induce reocclusion of blood vessels, aggravate the progression of AIS, and induce the occurrence of END [18]. Seo et al. [19] also confirmed that CRP is one of the important factors predicting the occurrence of END in AIS patients.

RETRACTED

This study found that patient age, OTT, NIHSS score, diabetes, hypertension, atrial fibrillation, infarct size, degree of carotid artery stenosis, and whether END occurred were statistically different between the poor prognosis group and the good prognosis group. Multivariate logistic analysis showed that age, NIHSS score, infarct size, degree of carotid artery stenosis, and END are all independent factors influencing the short-term prognosis of AIS patients after intravenous thrombolytic therapy. Among them, elderly patients are often accompanied by a variety of underlying diseases and varying degrees of vascular damage, so their prognosis is usually poor. The NIHSS score, the degree of carotid artery stenosis, and the infarct size may affect the short-term prognosis of AIS in a similar mechanism as inducing END. In addition, previous studies [20, 21] have also shown that END is closely related to the outcome of AIS patients and is an independent influencing factor of their short-term poor prognosis, similar to the results of this study. It should be pointed out that studies [22] reported that hypertension is one of the independent factors affecting the short-term poor prognosis of AIS patients. In this study, the number of patients with hypertension in the poor prognosis group was higher than that in the good prognosis group, but they did not enter the multivariate logistic analysis in the end. The possible reason is that blood pressure has a “U” relationship with the prognosis of AIS. Too low or too high can lead to insufficient blood reperfusion and poor prognosis in patients with AIS, and it is related to the circadian rhythm of blood pressure. The mechanism is complicated. The relationship between hypertension and the short-term prognosis of AIS is still inconclusive [23].

In summary, high NIHSS score, diabetes, atrial fibrillation, excessive infarct size, moderate to severe carotid artery stenosis, and elevated CRP are all risk factors for END after intravenous thrombolysis in AIS patients. Old age, high NIHSS score, large infarct size, moderate to severe carotid artery stenosis, and END are risk factors for poor short-term prognosis in patients with AIS after intravenous thrombolysis. Therefore, for AIS patients, it is necessary to do a good job of hospitalization assessment in time, a detailed understanding of the previous medical history, combined with imaging examinations, laboratory indicators, and early identification and early intervention of the occurrence of their END. At the same time, we pay attention to the prevention and treatment of END and try our best to improve the prognosis of AIS patients because of vigilant elderly AIS patients.

## Figures and Tables

**Table 1:** Univariate analysis of resulting in END of AIS patients (*n*, $\bar{x}$ ± *s*).

Influencing factors		END group (*N* = 71)	Non-END group (*N* = 141)	t/*χ*^2^ value	*P* value
Gender	Male	39	74	0.113	0.736
	Female	32	67		

Age (years)	≥60	43	64	4.349	0.037
	<60	28	77		

OTT (min)	210.45 ± 60.12	190.36 ± 70.43	2.055	0.041	
NIHSS score (points)	15.48 ± 3.37	13.16 ± 2.13	2.547	0.012	
Smoking	Yes	48	83	1.528	0.216
	No	23	58		

Drinking	Yes	37	69	0.191	0.662
	No	34	72		

Diabetes	Yes	18	19	4.623	0.032
	No	53	122		

Hypertension	Yes	32	42	4.854	0.028
	No	39	99		

Atrial fibrillation	Yes	21	23	5.052	0.025
	No	50	118		

TOAST classification	Large atherosclerosis type	39	30	4.883	0.027
	Arteriolar occlusion type	17	83		
	Psychogenic type	9	17		
	Clear other etiology types	4	5		
	Cryptogenic	2	6		

Infarct area (cm)	Diameter ≥3	41	52	8.350	0.004
	Diameter<3	30	89		

The degree of carotid stenosis	≥50%	29	37	4.697	0.030
	<50%	42	104		

Infarct site	Cortex	34	83	2.301	0.129
	Subcortical	37	58		

TC (mmol/L)		4.96 ± 1.24	4.57 ± 1.09	1.478	0.143
TG (mmol/L)		1.77 ± 1.89	1.91 ± 1.05	0.404	0.687
LDL-C (mmol/L)		3.15 ± 1.56	3.27 ± 1.14	0.374	0.709
HDL-C (*μ*mol/L)		17.86 ± 5.31	17.64 ± 4.32	0.376	0.707
UA (*μ*mol/L)		375.82 ± 154.66	363.39 ± 158.75	1.147	0.255
WBC (×109/L)		6.73 ± 1.66	6.18 ± 1.57	2.361	0.019
CRP (mg/L)		8.46 ± 2.17	6.39 ± 1.91	7.111	≤0.001
FIB (g/L)		3.22 ± 1.11	3.03 ± 0.91	1.331	0.185
D-D (mg/L)		3.32 ± 1.45	2.77 ± 1.26	2.850	0.005

RETRACTED

**Table 2:** Analysis of multiple factors affecting the appearance of END in AIS.

Influencing factors	B	SE	Wald's	Sig.	Exp (B)
Age	0.295	0.425	1.633	0.623	0.989
OTT	0.147	0.217	3.121	0.069	1.237
NIHSS score	0.275	0.287	3.339	0.013	1.845
Diabetes	0.213	0.245	3.549	0.048	1.721
Hypertension	0.276	0.189	7.014	0.079	1.341
Atrial fibrillation	0.194	0.158	7.771	0.034	1.786
The type of TOAST	0.188	0.207	4.388	0.081	1.643
Infarct size	0.254	0.356	2.004	0.041	1.639
The degree of carotid stenosis	0.311	0.247	5.098	0.022	2.145
WBC	0.268	0.199	6.543	0.088	1.246
CRP	0.273	0.299	3.054	0.029	2.237
D-D	0.185	0.217	3.929	0.063	1.377

**Table 3:** Single-factor analysis affecting the short-term prognosis of AIS patients (*n*, $\bar{x}$ ± *s*).

Influencing factors		Poor prognosis group (*N* = 85)	Good prognosis group (*N* = 127)	t/*χ*^2^ value	*P* value
Gender	Male	41	72	2.386	0.122
	Female	44	55		

Age (years)	≥60	54	53	9.678	0.002
	<60	31	74		

OTT(min)	218.34 ± 65.12	188.96 ± 70.43	3.067	0.002	
NIHSS score (points)	16.17 ± 1.18	14.22 ± 2.16	7.595	≤0.001	
Smoking	Yes	59	72	3.489	0.062
	No	26	55		

Drinking	Yes	41	65	0.176	0.674
	No	44	62		

Diabetes	Yes	21	16	5.181	0.023
	No	64	111		

Hypertension	Yes	38	36	5.998	0.014
	No	47	91		

Atrial fibrillation	Yes	25	19	6.466	0.011
	No	60	108		

TOAST classification	Large atherosclerosis type	32	37	2.342	0.129
	Arteriolar occlusion type	34	66		
	Psychogenic type	12	14		
	Clear other etiology types	3	6		
	Cryptogenic	4	4		

Infarct area (cm)	Diameter ≥3	49	44	10.941	0.001
	Diameter<3	36	83		

The degree of carotid stenosis	≥50%	35	31	6.677	0.010
	<50%	50	96		

Infarct site	Cortex	42	75	1.915	0.166
	Subcortical	43	52		

TC (mmol/L)	4.52 ± 1.18	4.77 ± 1.25	1.213	0.199	
TG (mmol/L)	1.84 ± 1.75	1.89 ± 1.34	0.679	0.688	
LDL-C(mmol/L)	3.29 ± 1.77	3.17 ± 1.24	0.464	0.794	
HDL-C (*μ*mol/L)	17.68 ± 4.21	17.95 ± 5.88	0.399	0.842	
UA (*μ*mol/L)	381.62 ± 154.36	361.79 ± 164.65	1.136	0.233	
WBC (×10^9^/L)	6.59 ± 1.37	6.88 ± 1.19	1.636	0.103	
CRP (mg/L)	7.92 ± 1.57	7.77 ± 1.81	0.623	0.534	
FIB (g/L)	3.46 ± 1.34	3.18 ± 1.31	1.511	0.132	
D-D (mg/L)	3.11 ± 1.19	3.24 ± 1.27	0.749	0.455	
END	Yes	40	31	11.727	0.001
	No	45	96		

RETRACTED

**Table 4:** Analysis of multiple factors affecting the short-term prognosis of AIS patients.

Influencing factors	B	SE	Wald's	Sig.	Exp (B)
Age	0.246	0.317	2.448	0.033	1.561
OTT	0.159	0.236	2.855	0.463	0.972
NIHSS score	0.276	0.198	7.040	0.026	1.768
Diabetes	0.236	0.278	3.054	0.069	1.843
Hypertension	0.274	0.185	7.671	0.093	1.571
Atrial fibrillation	0.217	0.166	7.875	0.123	1.576
Infarct size	0.236	0.312	2.219	0.046	0.989
The degree of carotid stenosis	0.311	0.247	4.752	0.022	2.145
END	0.216	0.179	6.741	0.006	2.832

## Data Availability

The data that are used or analyzed in the research can be obtained from the corresponding author according to reasonable requirements.
